The article "On the Visual Construction of Environmental Factors in Modern Art Works from the Perspective of Painting Art" was retracted in 2023. Reasons: signs of a paper mill; unreliable results or conclusions; concerns about the data; concerns about the peer review.

# On the Visual Construction of Environmental Factors in Modern Art Works from the Perspective of Painting Art

**DOI:** 10.1155/2022/5922048

**Published:** 2022-10-07

**Authors:** Shanshan Gong

**Affiliations:** School of Arts and Design, Xi'an University, Xi'an, Shaanxi 710065, China

## Abstract

Since the twenty-first century, with the continuous improvement of economic life, people have higher and higher requirements for life at present. Therefore, exploring better environmental art design has become a key concern of many people. This kind of environmental design can rely on the development of modern art in China. By analyzing the atmosphere of environmental factors and visual construction methods in modern art works, it can be integrated into the geographic positioning and map construction of slam in artificial intelligence. After analyzing the flavor of the times and visual construction of modern art, it is believed that SLAM algorithm can be combined with full convolution network FCN and superpixel CRF and can better estimate the position in many dynamic scenes. Therefore, we should explore in different ways, integrate the art culture in modern art works with modern social science and technology, and realize the modernization of environmental art design. It can be seen that the slam system formed by combining with the visual construction of environmental factors in modern art works is more suitable for people's life at the current stage.

## 1. Introduction

From the late Ming Dynasty to the Qianlong period of the Qing Dynasty, the development of relevant regional art schools and the interaction between the court and local artists facilitated and promoted the introduction of western modern art into the folk and the court to a certain extent [1]. This kind of introduction was mainly through missionaries and later gradually through commercial channels. The influence of art styles in different regions of Europe was also played in different situations where China and the West intersected. Through the fusion of the SLAM algorithm, the basic matrix is calculated through the IMU preintegration results, and the distance from the characteristic points to the epipolar line is calculated according to the basic matrix, and the points with large errors are eliminated. Finally, the random sample consistency algorithm is used to eliminate the mismatching points, which effectively improves the mismatching problem.

Since the seventeenth century, European perspective and copperplate have developed on the basis of modern mathematics and industry and Commerce [2, 3]. Because of their close relationship with the basic language of art, such as composition and sketch, they can be “internalized” into a more universal and civilian basic way of viewing and visual language communication, gradually breaking through the shackles of Baroque and the magnificent style of French Academy. However, in the seventeenth and eighteenth centuries, the western art contacted by the Chinese upper class and the intellectual class mostly belonged to the part related to missionaries and with court color. The new development of Western art modernity represented by the innovation of perspective and copper engraving was difficult to have a deep impact on Chinese local art. Even later, the influence of foreign art on the folk through commercial and other channels increased, leaving the initiative and systematic cognition of the local intellectual class; these influences often stayed at the external superficial level.

The development of modern factors of European art is also related to the growth and decline of different regions, national cultures, and corresponding art schools, and the development of art style schools is closely related to art education and communication. Starting from this idea, taking into account cultural geography and historical evolution, the following discusses the basic clues in the development and dissemination of style schools and modern visual methods in the early spread of western modern art in China [4].

Aiming at the problem that the 3D dense map constructed by the traditional slam system usually contains only low-level information such as color, depth, and brightness, this paper constructs an environmental semantic map based on the traditional 3D dense map, associates the 2D semantic labels in multiple frames, transfers them to the 3D point cloud through Bayesian update, and obtains a preliminary 3D semantic map [5]. On this basis, this paper proposes a global optimization algorithm of 3D semantic map based on high-order CRF. The algorithm establishes the high-order term of CRF through the spatio-temporal-consistent 3D superpixels, increases the constraint relationship between the point cloud and its 3D region, realizes the boundary consistency of the category of the point cloud in semantic segmentation, alleviates the influence of excessive smoothing caused by the binary term, and improves the segmentation accuracy. Experimental results show that this algorithm can obtain a globally consistent semantic map and effectively improve the semantic segmentation accuracy of a single frame image.

## 2. Literature Review

The early visual simultaneous localization and mapping (VSLAM) was achieved through filters. The widely used filter-based VSLAM is MonoSLAM proposed by davison3 in 2007 [6]. MonoSLAM is the first monocular real-time slam system based on feature point method. Its basic idea is as follows: extract Shi-Tomasi corners for each frame of image, assume that each corner follows Gaussian distribution, express its mean value and uncertainty through ellipse, and complete feature matching in projection ellipse. The mean and variance of the state vector are obtained by iterative updating. MonoSLAM only considers the state of the current frame and has nothing to do with the state of the previous frame, and the front end only tracks very sparse feature points, so the amount of calculation is small, which initially solves the problem of real-time. However, the error of the previous frame is transmitted to the next frame as a priori, and the error in the prior information cannot be eliminated, resulting in cumulative error. MonoSLAM is a milestone in the history of slam development, which has laid a solid foundation for the development of slam (as shown in Figure 1) [7, 8].

Wang proposed a semantic slam system based on deep learning and monocular visual slam in 2016. The system is combined with CNN on the basis of LSD-SLAM. It only performs semantic segmentation in key frames and selects adjacent frames to enhance the reconstruction effect. Therefore, it has good real-time performance and strong robustness in outdoor large scenes [9].

The 3D dense map constructed by the traditional visual slam system usually contains only low-level information, which cannot meet the intelligent requirements of robots. Based on the traditional three-dimensional dense map, this paper constructs the environmental semantic map and gradually transfers the two-dimensional semantic labels to the three-dimensional point cloud through Bayesian update. Aiming at the problem of fuzzy segmentation of object edges in 3D semantic map, a global optimization algorithm of 3D semantic map based on high-order conditional random field is proposed to optimize the semantic map and finally obtain a globally consistent semantic map (as shown in Figure 2) [10].

## 3. Atmosphere of Environmental Factors in Modern Art Works

### 3.1. Social Suffering

Looking at the modern history of the world, many countries have undergone major social changes. Among them, the most prominent is the gradual end of feudal society [11]. However, compared with many other countries, China's feudal society ended later. At the same time, China lags behind many countries in many aspects due to its long-term isolation from the outside world. Even after the end of the Qing Dynasty, Chinese society was still full of war and poverty, and people's lives had not been fundamentally improved. In the backward social environment, many Chinese artists expose social contradictions and criticize the dark phenomena in society through their works, to express their thoughts and feelings of longing for progress and calling for social change (see Figure 3) [12].

Printmaker Jiang Feng depicted a group of stevedores walking along the Huangpu River in the form of black-and-white woodcut in the woodcut “dock workers” [13]. Through the color change from black to white, people cannot help thinking of the scenes of tired workers who go out early and return late and work hard. The complex facial depiction highlights the workers' traumatic sense of vicissitudes in labor and clearly shows the author's deep sympathy for workers. As a common people group in the dark social environment, there were a considerable number of art works with the theme of workers at that time. Zhang Wang's work “injured head” depicts the image of a wounded worker. The roughness of the face is in sharp contrast to the firmness of the eyes, which makes people directly feel the valuable spirit of the characters' tenacious survival in suffering. At the same time, the bandaged eyes implied his miserable experience, reflecting the sharp social contradictions at that time.

In addition to printmaking, comics were also a common type of Chinese art in that period. Many cartoonists are good at creating satirical cartoons, attacking many negative phenomena in society and the difficulty of people's life with exaggerated and vivid nonrealistic techniques. The famous cartoonist Zhang Leping had the experience of being an apprentice in different places and also had a profound experience of the bitterness of the world in the difficult living environment. In his works, through the experience of the character “San Mao,” he showed the hardship and sadness of the people at the bottom of modern Chinese society in many ways, which aroused the sympathy of many people. However, grief is not the only thing in his works. In many comic strips, the characters are always exaggerated and lively. “San Mao,” as an urchin, also shows a lot of fun consistent with his age. This also highlights the valuable optimism of the people at the bottom represented by “San Mao” who are still strong in facing life after suffering discrimination and setbacks and also helps people alleviate their inner depression.

### 3.2. Resistance to Aggression

In the early twentieth century, China experienced many large-scale wars represented by the Second World War [14]. In the process of resisting Japanese aggression, China lost many resources and land, and countless innocent people died in the war. Facing the crisis of the country, many Chinese people also showed unprecedented unity. In addition to the army, the role of art works in the war cannot be ignored. Through their works, many artists express their strong feelings of resisting aggression and worrying about the country and the people, causing people to pay attention to the fate of the country (see Figure 4).

Long before the beginning of the war of resistance against Japan, Lu Xun, as a revolutionary, advocated new prints in China, believing that “when the revolution, prints were most widely used, although in a hurry, they could be done in an instant.” As Lu Xun expected, during the war, printmaking almost became the mainstay of Chinese art. Many artists directly publicized the anti-Japanese war in the form of prints, calling on people to defend and fight for the motherland. This is extremely valuable in an environment where painting tools are very scarce. Printmaker Li Shaoyan has left many works on the theme of the war of resistance against Japan. His works such as “landmine warfare” and “120th division in North China” vividly show the tenacity and heroism of the Chinese Army during the war of resistance against Japan, in sharp contrast to the enemy troops fleeing in haste in the picture, which not only reflects history, but also inspires all patriotic people.

While printmaking developed, other kinds of paintings also embodied their own role during the war. The famous painter Xu Beihong's masterpiece “Yu Gong moving mountains” was created during the most difficult period of the anti-Japanese war [15]. This work borrows the allusion of Yu Gong's removal of mountains, implies the importance of people's unity during the war of resistance against Japan, and appeals to the Chinese people to work together to win. It is a work of precious contemporary significance. During the war, the propaganda work of Chinese art never stopped. With the deepening of the war, the location of the Chinese art exhibition has shifted from the bustling downtown to the more remote countryside. This has given more people from rural areas the opportunity to appreciate revolutionary art and understand the environment of the times. Viewing art works does not require necessary skills such as literacy, which also highlights the strong tendency of Chinese art creators at that time to make art popular and folk.

## 4. Visual Construction in Modern Art Works

### 4.1. Regional Style Schools

Before the twentieth century, the “international style” in the Late Middle Ages was the last international style. Since then, the competition between European Nation States has even been reflected in the art activities of missionaries in China. The Netherlands has developed a unique populist style and commercial art and has launched commercial competition with both old and Protestant countries in the East. In the long-term confrontation between “pure art” of grand style and industrial and commercial art of citizen interest, the efforts to seek new unity even continued until the early twentieth century. Guo and Zhang got rid of the confrontation between salon art and handicraft and sought the unity of elite and mass, art, and technology. Modernist art in the twentieth century, especially the “international style” of architecture, can represent a new round of the pursuit of universality [16].

Tian and others “transported the gullies of Song people with the charm of popularity in the Yuan Dynasty,” which is based on professional painters and represents the trend of North-South integration [17]. Based on the enhancement of craftsmanship and visualization, the art in the early Qing Dynasty also showed a systematic and integrated trend. For example, the official sample system of porcelain in the Qing Dynasty reflects the management and systematic standardization of rival industries and also reflects the interest of scholars. The intervention of rival industries tends to be strengthened. The Qing emperor even supervised the process flow of ceramics and enamel. In the early Qing Dynasty, while strengthening the “pure art” to reflect the humanistic order, art also paid attention to its mutual penetration with craft categories. In the arts and crafts of the Ming and Qing Dynasties, the interaction between folk and official increased. In the Ming Dynasty, many painters and decorators were promoted to officials. With the development of China's hierarchy, from the enfeoffment of aristocracy to the military upstart and then to the imperial examination, the variable factors of social rank have increased. After the middle of the Ming Dynasty, the role of economic factors in social status increased, and China thus had more modern social factors. These are also what we should consider when we investigate the early spread of western modern art to China. Since the late Ming Dynasty, the regional shaping and cultural infiltration have also been interwoven with the efforts of art systematization.

Xu and Li believe that the Yangzhou Slender West Lake white tower, which was borrowed from the north in the late Qianlong period, “has left its original geographical background and removed its original religious significance.” These carefully crafted exhibits which can be regarded as local participation in a culture [18]. Astafiev and others used the extreme dramatic example of Zhang Dai's performance in Jinshan Temple in the middle of the night to illustrate that the cultural infiltration of Buddhist temples by the gentry in the late Ming Dynasty was almost unimaginable at any other time in Chinese history. He is not a devout believer, but expansively infiltrates religious places in the form of art. The expansionary expression of this “Baroque” artistic emotion, the dilution of religious doctrines, and the infiltration of cultural consciousness into regional space are also a reference for investigating the ideas of scholars on foreign cultures and religions, including Catholicism, since the end of the Ming Dynasty [19].

### 4.2. Development of Modern Visual Mode

Italian Renaissance art is complex. Poetic symbolic language and mathematical-based scientific language coexist with grand style and civic style, but poetic symbolic language and grand style later prevailed [20]. Russell pointed out that Renaissance Italians did not respect science except Da Vinci and others. After the eighteenth century, the industrial and commercial color in art, the interest of citizens, and the development of scientific visual language are related to some potential tendencies in the development of northern European culture. After getting rid of the guild with the help of the college, painting and sculpture art became “pure art,” and the handicraft category that used to belong to the guild is now facing the depreciation of “pure art” (in addition to perspective teachers, boss also has an identity as a printmaker regarded as a craftsman). Even Bauhaus in the early twentieth century needs to work hard to get rid of the influence of “salon art.” The classical perspective theory of pursuing magnificent style represented by LeBlanc and the perspective theory of emphasizing mathematics represented by boss extend to the East, represented by Nian Xiyao's “vision” and boss' book on the dissemination of Deszag theory imported from the Netherlands. Although the extent to which Japan can absorb Deszag's theory is still worth further discussion, Japan gradually began to learn western modern painting from the perspective of technology and service industry and commerce through books imported from the Netherlands (see Figure 5) [21].

At the same time, the folk painting formula reflects the confidential nature of similar guilds. This summary has not changed or even confirmed the social status and knowledge closeness of craftsmen [22]. In addition to social reasons, this is also determined by the internal nature of the organization and dissemination of Chinese visual art knowledge. In Europe, the formation of a subjective, objectified, and generalized visual way such as perspective is conducive to the potential systematization and generalization of visual art knowledge, just as the further development of perspective and the “internalization” of the visual way of print printing are reflected. In the Qianlong court, some Chinese and Western painters combined their brushwork for other purposes, but there were aesthetic inconsistencies. At the end of the Ming Dynasty, Dong Qichang's landscape contained irony. Some of the combined strokes in Zeng Jing's and Chen Hongshou's figure paintings, even if they contained realistic factors influenced by the west, and reflected and deepened the spiritual separation between the Literati's ideal and social reality through the comparison with the Literati's pen and ink. Pu Andi linked the visual art in the late Ming Dynasty with the “irony” in the “four wonderful books” of Literati novels. Behind the self-consciousness embodied in this irony is still the Confucian ideal, which is different from the civil culture since the European Renaissance [23].

## 5. Analysis of Visual Fusion Algorithm Based on Art Works

### 5.1. Superpixel-Based Edge Optimization

The superpixel segmentation algorithm can be divided into graph-based superpixel segmentation algorithm and gradient descent-based superpixel segmentation algorithm [24]. The graph-based superpixel segmentation algorithm takes pixels as the basic nodes in the graph, gives different weights to the edges according to the similarity between adjacent pixels, establishes an undirected graph objective function, and minimizes this objective function to obtain superpixels. The superpixel segmentation algorithm based on gradient descent randomly initializes a cluster center and makes the cluster center tend to be stable by gradient descent method. At present, superpixel segmentation algorithm is widely used in the field of computer vision. Considering that the superpixel can better fit the edge of the object and establish a constraint relationship between the pixels of different objects, this paper uses the superpixel to optimize the semantic rough segmentation image extracted from the front end to improve the segmentation accuracy of the object edge (as shown in Figure 6) [25].

SLIC algorithm is a local clustering algorithm based on *k*-means. Its main idea is not complex, its implementation is relatively simple, and its calculation efficiency is high. It can better maintain the edge information of objects and generate superpixels of various sizes to adapt to the system. It is widely used in image preprocessing in image processing. SLIC algorithm clusters pixels through five 14 dimensional feature vectors, which include two-dimensional spatial position information represented by *x* and *y* and three-dimensional color information represented by CIELAB (see Figure 7).

Its main ideas are as follows.

The first step is to initialize the seed points. The initial seed points are *C*, the number of pre segmented superpixels is *K*, and the number of pixels is *n*. The image is divided into grids, each grid contains *N*/*K* pixels, and the step size between seed points is:

(1) $$\begin{array}{c} S=\sqrt{\frac{N}{K}}. \end{array}$$

The second step is clustering. Sobel filtering is used for the pixels in the neighborhood of the initialized seed point *n*∗*n*, and the point with the smallest gradient is selected as the new seed point to avoid the seed point falling to the edge. After reselecting the seed points, calculate the similarity between the seed points and the pixels in the 2*S*∗2*S* neighborhood. *M* is the balance parameter, *d*_*c*_ is the color similarity between the seed points and the pixels in the neighborhood, and *d*_1_ is the position similarity between the seed points and the pixels in the neighborhood and is the similarity measure after combining the distance between the two:

(2) $$\begin{array}{c} d_{c}=\sqrt{\left(l_{j}-l_{i}\right)2+{\left(a_{j}-a_{i}\right)}^{²}+{\left(b_{j}-b_{i}\right)}^{²}},\\ d_{1}=\sqrt{{\left(x_{j}-x_{i}\right)}^{²}+{\left(y_{j}-y_{i}\right)}^{²}},\\ D=d_{c}+\frac{m}{s}\;d_{1}. \end{array}$$

Then, for iterative optimization, the second step can be repeated until each seed is no longer changed. Finally, relatively isolated points are removed to enhance the connectivity of the whole segmented image. So far, the superpixel segmentation of the image is completed. After the completion of image semantic rough segmentation and image superpixel segmentation, the results of the two will be combined. The effect of image edge optimization depends on the effect of the combination of superpixel edge and image semantic rough segmentation (as shown in Figure 8).

If the segmentation of superpixels and semantics is accurate enough, the pixels in each superpixel belong to the same category, but the segmentation of semantic rough segmentation at the edge of the object is relatively fuzzy, which cannot guarantee error free segmentation. Due to the error of semantic segmentation, a superpixel may contain multiple categories of pixels, which can be passed through:

(3) $$\begin{array}{c} \;P=\frac{1}{K}\overset{K}{\underset{i=1}{\sum }}p_{i}. \end{array}$$

where *K* represents the number of pixels in the superpixel block; *p*_*i*_ represents the probability distribution of the category of the *i*th pixel obtained from FCN and then calculates the entropy value corresponding to each superpixel. If the segmentation result is more accurate, and the pixels in the superpixel contain only one category, the corresponding entropy value is small, and there is no need to re segment. If there is an error in semantic segmentation in a superpixel, the pixels in the superpixel contain multiple categories. If two different probability distributions are fused together, the corresponding entropy value is large and need to be resegmented (as shown in Figure 9).

### 5.2. Feature Extraction and Tracking

Visual odometer can be divided into odometer based on descriptor feature matching and odometer based on optical flow tracking according to different implementation methods. For odometer based on descriptor feature matching, first extract feature points from the image, then calculate the descriptor, and then match the features according to the descriptor. This method can obtain more accurate data association, but the process of feature extraction and matching requires a lot of computing resources, and the real-time performance is poor. The real-time performance of optical flow tracking is good, but there are also some limitations. The premise of optical flow tracking is that the motion between two consecutive frames is small. If the optical flow method is no longer applicable in the fast-moving scene, the optical flow method can be used to track feature points, which can combine the advantages of both. To solve the above problems, this paper introduces a multiscale optical flow tracking algorithm based on orb characteristics and LK optical flow method (as shown in Figure 10).

The traditional slam system completes pose estimation under the assumption that the scene is fixed, ignoring the impact of dynamic objects in the scene on pose estimation. Aiming at the problem that dynamic objects reduce the accuracy of pose estimation of slam system, this section proposes a dynamic feature point detection algorithm based on semantic information and polar constraint. The dynamic feature points in the scene are eliminated through the relationship between semantic information and polar constraints, so that the slam system can build geometric position constraints according to the static feature points in the scene and solve the relative motion of the camera (as shown in Figure 11).

### 5.3. Optical Flow Tracking

When the camera moves in the scene, the acquired image changes, corresponding to the change of optical flow field in the image. Optical flow is a method to describe the movement of pixels in the image with time. Optical flow method is divided into sparse optical flow method and dense optical flow method. Dense optical flow tracks all pixels in the image, while sparse optical flow tracks some pixels in the image. The extracted ORB feature points are evenly distributed on the image, which can better reflect the transformation relationship between the two images. Therefore, using sparse optical flow can well meet the requirements of the system.

LK optical flow algorithm is a classic sparse optical flow tracking algorithm, which is constructed by the following assumptions.

First, the assumption of gray level invariance, that is, the pixels of the same spatial point in any frame of the image remain gray level invariable.

Second, “small motion” hypothesis, that is, the camera is moving slowly, that is, the transformation between two frames of images is small.

Third, the neighborhood consistency assumption, that is, a pixel and its neighborhood pixels have consistent motion (as shown in Figure 12).

When optical flow tracking is performed between two consecutive images, ORB feature points are first extracted from the previous image, and the coordinate values of these ORB feature points are used as the initial values of the pyramid optical flow algorithm. Then, the coordinates of these feature points in the current frame are obtained through the pyramid optical flow algorithm. The difference between the two coordinates is the optical flow value corresponding to the feature point. Calculate the optical flow value of all feature points and take the mean value, that is, the optical flow between two consecutive frames of images (as shown in Figure 13).

### 5.4. Dynamic Feature Removal

After the feature point tracking between two consecutive frames is completed, it is necessary to build a geometric constraint relationship for the matching feature points between two consecutive frames to recover the relative motion between the two frames. The traditional slam system estimates pose under the assumption that the scene is fixed, ignoring the impact of dynamic objects in the scene on pose estimation. The feature points on dynamic objects will seriously affect the accuracy of pose estimation. To solve the above problems, a dynamic feature point detection algorithm based on semantic information and polar constraints is proposed. The potential moving object is obtained through the semantic segmentation results, and the feature points on the object are judged whether they are dynamic feature points. If they are dynamic feature points, they are eliminated, and if they are static feature points, they are retained (as shown in Figure 14).

Finally, the position and attitude of the camera are estimated by using the dynamically eliminated feature points, which improves the robustness of the SLAM system in the dynamic environment. Therefore, the essence of epipolar geometry is the geometric constraint relationship between the image plane and the plane bundle with the baseline as the axis. The epipolar constraint relationship can be established between the corresponding points in different frames at the same spatial point (as shown in Figure 15), and it can also be carried out through triangle measurement (as shown in Figure 16).

The two pixels *P* are the projection points of *P* in the two images. The plane composed of *O* and *P* is the polar plane and intersects with the *L* polar line, and the intersection *e* of the two images is the pole. In the process of elimination, relevant standard processes should be followed (as shown in Figure 17).

### 5.5. IMU Motion Model and Preintegration

In the visual inertial odometer, the sampling frequency of IMU is much higher than that of the camera. The sampling frequency of the camera is 20~30 Hz, and the sampling frequency of IMU is 200 Hz or even higher. In the timing relationship between IMU sampling frequency and camera sampling frequency (as shown in Figure 18), therefore, there are often many IMU measurements between two consecutive frames of images. Correct processing of IMU data between two frames of images is a crucial step in the visual inertial odometer. IMU preintegration can effectively fuse high-frequency IMU data with low-frequency image data, and is widely used in visual inertial odometer. The main idea of IMU preintegration is to integrate the IMU measurements between two consecutive frames into a relative motion constraint only related to the IMU measurements. When the state quantity is iteratively updated, the integral value is approximated by first-order Taylor, to prevent repeated calculation.

The visual inertia joint initialization is completed on the basis of obtaining the visual initialization results and IMU preintegration results, so the method can design the visual initialization part, and the accurate visual initialization results can provide accurate parameters for the visual inertia initialization (as shown in Figures 19 and 20) for the overall process.

## 6. Conclusion

Although the social environment in China in the early twentieth century was very bad, it failed to prevent Chinese artists from exploring art, and countless setbacks eventually became the source of inspiration for artists. Aiming at some defects of the traditional SLAM algorithm, this paper integrates the environmental factors and visual construction in different periods, puts forward some improvement schemes, integrates the semantic information into the slam system, and preliminarily achieves the expected goal. Semantic reprojection error can be introduced to strengthen the constraints of semantics on pose estimation, so as to improve the accuracy of pose estimation. Slam system obtains a large number of globally geometrically consistent image information, which can provide some support for deep learning model training.

## Figures and Tables

**Figure 1:** Frame motion estimation block diagram based on semantic information.

**Figure 2:** Semantic segmentation system diagram.

**Figure 3:** The timeline of modern China.

**Figure 4:** China's anti-Japanese war route.

**Figure 5:** Modern world development.

**Figure 6:** Block diagram of edge optimization based on superpixels.

**Figure 7:** SLIC algorithm clustering.

**Figure 8:** Image semantic separation and combination process.

**Figure 9:** Repartition cycle.

**Figure 10:** Multiscale light tracking.

**Figure 11:** Dynamic feature elimination algorithm.

**Figure 12:** Optical flow tracking.

**Figure 13:** Pyramid optical flow algorithm under ORB feature.

**Figure 14:** Retention of each static point.

**Figure 15:** Polar geometry diagram.

**Figure 16:** Triangle measurement diagram.

**Figure 17:** Dynamic feature point removal process.

**Figure 18:** Camera timing of IMU.

**Figure 19:** Visual initialization process.

**Figure 20:** Overall process.

## Data Availability

The labeled dataset used to support the findings of this study is available from the corresponding author upon request.
